RETRACTED

# Long non-coding RNA HIF1A-AS2 facilitates adipose-derived stem cells (ASCs) osteogenic differentiation through miR-665/IL6 axis via PI3K/Akt signaling pathway

**DOI:** 10.1186/s13287-018-1082-z

**Published:** 2018-12-13

**Authors:** Ruoyu Wu, Jihao Ruan, Yongjin Sun, Mengyu Liu, Zhuang Sha, Cunyi Fan, Qingkai Wu

**Affiliations:** 1 Institute of Microsurgery on Extremities, Shanghai Jiao Tong University Affiliated Sixth People’s Hospital, Shanghai, 200233 China; 2 Department of Orthopaedics, Shanghai Jiao Tong University Affiliated Sixth People’s Hospital, No.600 Yishan Road, Xuhui District, Shanghai, 200233 China; 3 Department of Obstetrics and Gynecology, Shanghai Jiao Tong University Affiliated Sixth People’s Hospital, Shanghai, 200233 China; 4 Institute of Nervous System Diseases, Xuzhou Medical University, Xuzhou, 221004 Jiangsu China

**Keywords:** HIF1A-AS2, miR-665, IL6, ASC, Osteogenic differentiation

## Abstract

**Background:**

This study was aimed to investigate the role and specific molecular mechanism of HIF1A-AS2/miR-665/IL6 axis in regulating osteogenic differentiation of adipose-derived stem cells (ASCs) via the PI3K/Akt signaling pathway.

**Methods:**

RNAs’ expression profile in normal/osteogenic differentiation-induced ASCs (osteogenic group) was from the Gene Expression Omnibus database. The analysis was carried out using Bioconductor of R. Gene Set Enrichment Analysis and Kyoto Encyclopedia of Genes and Genomes dataset were applied to identify up- and downregulated signaling pathways. Co-expression network of specific lncRNAs and mRNAs was structured by Cytoscape, while binding sites amongst lncRNA, mRNA, and miRNA were predicted by TargetScan and miRanda. ASCs were derived from human adipose tissue and were authenticated by flow cytometry. ASC cell function was surveyed by alizarin red and alkaline phosphatase (ALP) staining. Molecular mechanism of HIF1A-AS2/miR-665/IL6 axis was investigated by RNAi, cell transfection, western blot, and qRT-PCR. RNA target relationships were validated by dual-luciferase assay.

**Results:**

HIF1A-AS2 and IL6 were highly expressed while miR-665 was lowly expressed in induced ASCs. HIF1A-AS2 and IL6 improved the expression level of osteoblast markers Runx2, Osterix, and Osteocalcin and also accelerated the formation of calcium nodule and ALP activity, yet miR-665 had opposite effects. HIF1A-AS2 directly targeted miR-665, whereas miR-665 repressed IL6 expression. Moreover, the HIF1A-AS2/miR-665/IL6 regulating axis activated the PI3K/Akt signaling pathway.

**Conclusions:**

LncRNA HIF1A-AS2 could sponge miR-665 and hence upregulate IL6, activate the PI3K/Akt signaling pathway, and ultimately promote ASC osteogenic differentiation.

RETRACTED

**Electronic supplementary material:**

The online version of this article (10.1186/s13287-018-1082-z) contains supplementary material, which is available to authorized users.

## Background

The human skeleton is remodeling continuously throughout adult stage [1]. But on the condition of osteoporosis or severe traumatism such as fractures, the body usually loses bone mass and bone strength and suffers deficits in bone density and quality [2]. Although bone marrow mesenchymal stem cells (BMSCs) can differentiate into osteoblasts, the proliferative capability and osteogenic differentiation ability of BMSCs decrease with age [3, 4], the supply of such autologous stem cells is also limited [5]. As a potential alternative source, adipose-derived stem cells (ASCs), which is a kind of multipotential mesenchymal stem cell (MSC) capable of bone regeneration and reconstruction [6], have aroused interest of researchers on account of their widespread and abundance storage, easy access, and low-level pain/harm extraction [2]. ASCs are of great importance to the exploration of novel autologous therapies.

Long noncoding RNAs (lncRNAs) were found as a novel subset of non-coding RNAs, those which have over 200 nucleotides. Evidence showed that lncRNAs were related to multiple physiological and pathological processes by diverse mechanisms [7]. Recent studies indicated that some lncRNAs played a role in regulating osteogenic differentiation of stem cells [8], usually as competing endogenous RNA (ceRNA) which sponged at microRNAs (miRNAs), by which they regulated the expression of downstream messenger RNA (mRNA) [9]. HIF1A-AS2 is a kind of lncRNA which facilitates several cancers, such as colorectal cancer, bladder cancer, and glioblastoma [10–12]; it is considered as a diagnostic biomarker of the development in differentiation between diverse breast cancer types [13], as well as an influence on other processes including HUVEC angiogenesis [14]. A recent study revealed that HIF1A-AS1 and HIF1A-AS2 played a role in regulating hypoxia-inducible factor-1α (HIF-1α) and further affected periodontal ligament cell (PDLC) osteogenic differentiation [15]. But the effect of HIF1A-AS2 on ASC osteogenic differentiation still needs more exploration. Up to now, research on the relationship between HIF1A-AS2 and ASC osteogenic differentiation is very scarce, leaving us an ample room to explore and an arduous task to fulfill.

MicroRNAs (miRNAs) are clustered as single-stranded, highly conserved, non-coding RNA molecules, which regulate target gene expression by establishing direct interaction with homologous mRNA target 3′-untranslated regions (3′UTR) [16]. Several miRNAs have been confirmed to have important roles in skeletal development and disorders [17, 18], and the expression of some critical miRNAs also reflected the progress of bone-related diseases [19, 20]. According to a previous report, miR-665 took part in regulating carcinoma cell migration, invasion, and proliferation [21] and influenced the cell cycle through targeting mRNAs [22]. In terms of ASCs, some specific miRNAs also referred to an osteogenic differentiation process [23]. MiR-665 was reported functioning as a repressor of odontoblast osteogenic differentiation and mineralization [24]. It was of great significance to investigate the function of miR-665 in an ASC osteogenic differentiation process. In this research, we focus on the regulating mechanism of miR-665, regarding it as a bridge connecting lncRNA and mRNA. Interleukin-6 (IL6) with IL6 receptor (IL6R) plays a crucial part in the tissue regeneration in vivo, especially bone metabolism [25]. It was observed related to osteogenic differentiation of MSCs according to recent reports [26, 27]. IL6 can combine miRNAs [28], transmit the information to the signaling pathway PI3K/Akt which contains IL6 receptor, and promote osteogenic differentiation. It is worth noting that IL6 can also regulate the differentiation functions of ASCs [29]. Bakhit et al. revealed for the first time that SrRn promoted proliferation and odonto-/osteogenic differentiation/mineralization of methylene diphosphonates via PI3K/Akt signaling activated by CaSR in vitro; mineralized tissue forms from the dental pulp in vivo [30]. PI3K/Akt played a role in aortic valve interstitial cell (AVIC) inflammation and calcification promoted by IFN-α [31]. A growing number of studies revealed the possibility that the PI3K/Akt pathway affects osteogenic differentiation, but the effect of the PI3K/Akt pathway in ASC osteogenic differentiation remains to be studied.

RETRACTED

In our study, we compared the expression of lncRNAs and mRNAs between induced ASCs and undifferentiated ASCs and found the intersectional miRNA of lncRNA, mRNA, and the signaling pathway. According to bioinformatics analysis results, experiments were designed to explore the specific regulatory mechanism of the HIF1A-AS2/miR-665/IL6 chain which targeted the PI3K/Akt signaling pathway in the process of ASC osteogenic differentiation. This exploration may provide a primary foundation for future investigation of osteogenic differentiation and theories of bone-related diseases, contributing to the discovery of new therapeutic targets for illness and innovative skeleton modeling methods.

## Methods

### Bioinformatics analysis

The total RNA expression profile of obtained adipose-derived stem cells was from the Gene Expression Omnibus (GEO) database (GSE89330). We filtered lncRNAs and mRNAs which were differentially expressed by R version 3.4.1 (https://www.r-project.org/) with Limma. The criteria for DEGs were based on |fold change| > 2 combined with adjusted *P* value less than 0.05, and the results were exhibited as heatmaps.

Gene Set Enrichment Analysis (GSEA) (http://software.broadinstitute.org/gsea) and pathway gene set Kyoto Encyclopedia of Genes and Genomes (KEGG) (https://www.kegg.jp/kegg/) were used to implement gene set enrichment analysis. The data of mRNA involved in pathways was from KEGG and is showed in Additional file 1: Table S1. According to a report of GSEA, the joyplot and dotplot of highest up- or downregulated signaling pathways (adjusted *P* value < 0.05) were depicted.

Cytoscape version 3.6.0 (http://www.cytoscape.org/) was used to construct co-expression network of differentially expressed lncRNAs and mRNAs. Node and edge files were generated by R with the filtering condition of adjusted *P* value < 0.05 and threshold > 0.7.

Prediction of lncRNA and miRNA/miRNA and mRNA binding sites was carried out using the miRcode (http://www.mircode.org/) and TargetScan (http://www.targetscan.org/vert_71/) databases. The relationship between mRNA and the pathway/miRNA and pathway was investigated by String (https://string-db.org/) or DIANA Tools (http://diana.imis.athena-innovation.gr/DianaTools).

### Tissue specimens

Human ASCs were collected from 10 patients (5 males, 5 females) whose subcutaneous fat was taken by liposuction. The operation was conducted at Shanghai Jiao Tong University Affiliated Sixth People’s Hospital. All of our participants have signed informed consents, and experiments have been authorized by the ethics committee of Shanghai Jiao Tong University Affiliated Sixth People’s Hospital.

### Cell isolation and culture

Disinfected adipose tissues with 75% ethanol were rinsed by PBS for three times. Adipose tissue was cut into small fragments (< 5 mm) using a razor blade and digested by collagenase type II (0.1 mg/mL) (Sigma-Aldrich, St. Louis, MO, USA) for 60 min at 37 °C. We transferred the liquid into a centrifuge tube and did low-speed centrifugation at 800 r/min × 10 min. Suspension cells were filtrated by a 70-μm-diameter cell filter (BD Falcon, San Jose, CA, USA) and then were cultivated in low-glucose DMEM (Gibco, Grand Island, NY, USA) with 10% fetal bovine serum (FBS, Gibco) and 1% penicillin at 5% CO_2_ and 37 °C. On the next day, the unattached cells were removed and then ASCs were collected, washed thrice, and used for subsequent experiments.

To implement dual-luciferase assay, human embryo kidney cell line HEK-293 was purchased from BeNa Culture Collection (Beijing, China) and cultivated in high-glucose DMEM (Gibco) with 10% FBS.

RETRACTED

### Osteogenic induction

For osteogenic induction, ASCs were seeded at a density of 2.0 × 10^5^ cells/well into 12-well plates with routine medium. When cells reached 80–90% confluence, the medium was changed (contained 10% FBS, 50 μg/mL l-ascorbic acid, and 10 mM β-glycerophosphate), and cells were grown in osteogenic induction medium with the StemPro™ Osteogenesis Differentiation Kit (Gibco). The osteogenic induction medium was replaced every 3 days.

### Flow cytometry

CD29, CD31, CD44, and CD45 were selected to identify the isolated ASCs. CD29 and CD44 were primary stable positive markers of ASCs while CD31 and CD45 were primary negative markers of ASCs [32]. Additional 1 × 10^6^ cells were respectively incubated with PE-conjugated mouse antibody against CD31 (ab233642, 4 μL, Abcam), FITC-conjugated mouse antibody against CD29 (ab21845, 1.5 μL, Abcam), FITC-conjugated mouse antibody against CD44 (ab27285, 10 μL, Abcam), and PE-conjugated mouse antibody against CD45 (ab155385, 5 μL, Abcam) and isotype-matched control IgG (ab154450, 0.1 μg, Abcam). Flow cytometry was conducted by a FACSCanto™ II Flow Cytometer (BD Biosciences, San Jose, CA, USA).

### Cell transfection

AgomiR-665, antagomiR-665, pcDNA3.1-HIF1A-AS2, pcDNA3.1-sh-HIF1A-AS2 (sh-HIF1A-AS2), pcDNA3.1-IL6, pcDNA3.1-sh-IL6 (sh-IL6), and their respectively negative control (NC) came from GenePharma (Shanghai, China). 7.5 μL Lipofectamine 3000 (Invitrogen, Carlsbad, CA, USA) and 5 μg transfection object were respectively diluted by 250 μL serum-free DMEM with high glucose and incubated for 5 min in a room temperature environment. Then, pre-mixed solution was added into 2 × 10^5^ exponential phased ASCs which were inoculated into six-well plates and incubated for 48 h at 37 °C and 5% CO_2_. Puromycin was used to filter stabilized transfected cells.

### qRT-PCR

RNAs of ASCs were extracted using a TRIzol reagent (Invitrogen) and then reverse transcribed to cDNA using a SuperScript™ III Reverse Transcriptase Kit (Invitrogen) (for lncRNA and mRNA reverse transcription) and miRCURY LNA RT Kit (Qiagen, Duesseldorf, Germany) (for miRNA reverse transcription). qRT-PCR was conducted by a LightCycler 480 PCR System (Roche, Rotkreuz, Switzerland) using SYBR Green qPCR Master Mix (Takara, Tokyo, Japan). Relative expression of RNAs was calculated by a 2^−ΔΔCt^ method. Meanwhile, GAPDH was brought in as internal reference. PCR primers were synthesized by Sangon Biotech (Shanghai, China), and sequence information is exhibited in Table 1.

RETRACTED

**Table 1:** Primer sequences for qRT-PCR

Gene	Forward primer 5′–3′	Reverse primer 5′–3′
HIF1A-AS2	AGATCTGTGGCTCAGTTCCTTT	AATCACTATGAATCCCTGCACCT
miR-665	ACCAGGAGGCTGAGGCCCCT	Involved in the kit
IL6	TCAATATTAGAGTCTCAACCCCCA	GAGAAGGCAACTGGACCGAA
Runx2	CCTTCAAGGTGGTAGCCCTC	CCCTAAATCACTGAGGCGGT
Osterix (SP7)	AGACCTCCAGAGAGGAGAGAC	GGGGACTGGAGCCATAGTGA
Osteocalcin	AATAGCCCTGGCAGATTCCC	CTCTCATGGTGTCTCGGTGG
GAPDH	GACAGTCAGCCGCATCTTCT	GCGCCCAATACGACCAAATC

### Western blot

Proteins were leached by RIPA lysis buffer (Beyotime, Shanghai, China) and quantified by an Enhanced BCA Protein Assay Kit (Beyotime). Total 20 μg protein was split up by SDS-PAGE and transferred to PVDF membranes (Beyotime). Blocked by 5% concentration of bovine serum albumin (BSA, Sigma-Aldrich) at 37 °C for 0.5 h, the membranes were cultivated with primary antibodies at 4 °C overnight (using GAPDH as internal reference). Then, secondary antibody was added and the culture continued at room temperature for another 1 h. Washed three times by TBST, HRP-labeled proteins were introduced by BeyoECL Star Kit (Beyotime) and filmed. The primary antibodies were as follows: rabbit anti-IL6 (ab6672, 1:2000, Abcam, Cambridge, MA, USA), rabbit anti-IL6R (ab128008, 1:500), rabbit anti-pan-Akt (ab8805, 1:500), rabbit anti-pan-Akt (phospho T308) (ab38449, 1:500), and rabbit anti--GAPDH (ab181603, 1:10000). The secondary antibody was HRPlabeled goat anti-rabbit IgG (ab205718, 1:2000).

### Dual-luciferase reporter gene assay

HEK-293 cells were seeded into 12-well plates and cultured until the confluence of cells reached 80–90%. PCR was used to amplify the 3′UTR segments of the HIF1A-AS2 sequence and IL6 mRNA sequence containing the predicted miR-665 binding sites. The direct binding sites of miR-665 to HIF1A-AS2/IL6 were confirmed by miRCode or TargetScan. 3′UTR of HIF1A-AS2 or IL6 wild type (wt)/mutant type (mut) PmirGLO vectors (Promega, Madison, WI, USA) were built by an XL Site-directed Mutagenesis Kit (Qiagen). According to the manufacturer’s instructions, cells were transiently co-transfected with 0.2 μg HIF1A-AS2/IL6 3′UTR or HIF1A-AS2/IL6 3′UTR mutant reporter plasmids together with 100 nmol/L miR-665 or miR-NC using Lipofectamine™ 3000 (Invitrogen). Corresponding luciferase activity was evaluated by a Dual-luciferase Reporter Assay Kit (Promega) 48 h after transfection conforming to the manufacturer’s direction.

### Alizarin red staining

Alizarin red staining was conducted 21 days after the osteoblastic induction. The cells that were cultured on 12-well plates thrice were fixated with 4% paraformaldehyde for 30 min and stained with 1% alizarin red S solution (pH = 8.4) (Sigma-Aldrich) for 5 min. Later, they were washed by PBS again and were filmed under an optical microscope (Olympus, Tokyo, Japan). To quantify matrix mineralization, alizarin red-stained cultures were incubated in 100 mM cetylpyridinium chloride for 1 h at room temperature to solubilize calcium-bound alizarin red, the absorbance of which was measured at 570 nm and normalized to the cells without any treatment.

RETRACTED

### Alkaline phosphatase staining

Fourteen days after osteogenic induction, a BCIP/NBT Alkaline Phosphatase Color Development Kit (Beyotime) was used to perform alkaline phosphatase (ALP) staining. The cells cultured in 12-well plates were rinsed three times by PBS and fixated for 30 min using 4% paraformaldehyde. Next, BCIP/NBT ALP staining buffer was added and cells were cultivated (room temperature, 2 h) in a darkroom. After that, cells with ddH_2_O were rinsed and filmed under an optical microscope. The absorbance at 405 nm of each well was measured with a microplate reader according to the manufacturer’s instruction.

### Statistical analysis

All of the experiments were done repetitively at least three times. Using GraphPad Prism version 6.0 (GraphPad Software, La Jolla, CA, USA), we collected the data and visualized their mean ± standard deviation (SD). The difference between two groups was compared using Student’s *t* test, and comparison amongst three groups or above was done by one-way ANOVA. *P* < 0.05 indicated statistical significance.

## Results

### Differently expressed lncRNAs and mRNAs in induced ASCs

Expression data of GSE89330 was analyzed by R package Limma. Based on the screening conditions that log_2_ (fold change) > 1 and adjusted *P* value < 0.05, 985 lncRNAs (507 down, 478 up) and 2535 mRNAs (1384 down, 1151 up) were screened out which were differently expressed in induced ASCs. We chose top-30 up- and downregulated lncRNAs and mRNAs to draw the heatmaps (Fig. 1a, b).

**Fig. 1:** Differentially expressed lncRNAs and mRNAs in normal/induced ASCs. **a** Heatmap of top-30 up- or downregulated lncRNAs in normal/induced ASCs. **b** Heatmap of top-30 up- or downregulated mRNAs in normal/induced ASCs

### KEGG pathway enrichment analysis

GSEA was performed using data profile of differentially expressed mRNAs screened out by R and KEGG dataset. Top-7 up- and downregulated signaling pathways are shown in Fig. 2a. Herein, we discovered that the PI3K/Akt signaling pathway was notably activated in induced ASCs (Fig. 2b). Pathway expressions were also visualized in the form of a joyplot (Fig. 2c) and dotplot (Fig. 2d); the results showed hepatitis B, hepatitis C, cAMP, drug metabolism cytochrome P450, measles, JAK/STAT, and PI3K/Akt, and tyrosine metabolism signaling pathways were significantly activated while protein processing in endoplasmic reticulum, lysosome, and rheumatoid arthritis, epithelial cell signaling in helicobacter pylori infection, and phagosome signaling pathways were conspicuously suppressed. All of these results suggested the PI3K/Akt signaling pathway was activated in induced ASCs.

RETRACTED

**Fig. 2:** Pathway enrichment analysis based on differentially expressed mRNAs. **a** GSEA plot for top-7 upregulated signaling pathways in normal/induced ASCs. **b** GSEA report for the PI3K/Akt signaling pathway showed that it was upregulated in induced ASCs. **c** Joyplot of GSEA reports showed that the PI3K/Akt signaling pathway was upregulated. **d** Dotplot of GSEA reports showed that the PI3K/Akt signaling pathway was upregulated

### Construct co-expression network and filter miRNAs

We intersected differentially expressed mRNAs in osteogenesis ASCs and mRNAs involved in the PI3K/Akt signaling pathway. A related mRNA IL6 was found remarkably highly expressed in osteogenesis ASCs (log_2_ (fold change) = 3.302) by Limma package. According to String and KEGG analyses (Fig. 3a), we affirmed that IL6 could activate protein IL6R. Moreover, to verify a possible relationship between IL6 and lncRNAs, we used R and Cytoscape to build a co-expression network between differentially expressed lncRNAs and mRNAs according to the screening condition in which Pearson correlation coefficient > 0.7 and *P* < 0.05 (Fig. 3b). The network indicated that IL6 was in co-expression with lncRNAs HIF1A-AS2. Hence, we proposed a hypothesis that HIF1A-AS2 might regulate IL6 by sponging miRNAs. Using TargetScan and miRcode databases, we filtered all miRNAs that would bind to HIF1A-AS2 or IL6 3′UTR. DIANA Tools was applied to search miRNAs related to the PI3K/Akt signaling pathway. MiR-665 was figured as a link between HIF1A-AS2 and IL6 (Fig. 3c), and binding sites were predicted for each relationship (Fig. 3d). Therefore, the following experiments were designed to explore the HIF1A-AS2/miR-665/IL6 axis.

**Fig. 3:** Analysis of lncRNA/miRNA/mRNA axis. **a** String: downstream proteins of IL6, including IL6R. **b** Co-expression network of lncRNA/mRNA built by Cytoscape. HIF1A-AS2 and IL6 had a positive correlation. **c** Venn diagram of miRNA binding HIF1A-AS2/IL6 and miRNA involved in the PI3K/Akt signaling pathway. MiR-665 was screened out. **d** Predicted binding sites between miR-665 and HIF1A-AS2/IL6 3′UTR

### Identification of ASCs and HIF1A-AS2 expression in ASCs

Flow cytometry was performed to identify ASC surface markers including CD29, CD31, CD44, and CD45 (Fig. 4a), and the results showed that 90.5% of ASCs expressed CD29, 82.3% expressed CD44, 9.4% expressed CD45, and 8.6% expressed CD31, making clear the identity of isolated ASCs. Then, we carried out osteogenic induction and identified HIF1A-AS2 expression in normal/induced ASCs using qRT-PCR at time nodes of 1, 2, or 3 weeks. It is shown that HIF1A-AS2 expression in induced ASCs was remarkably higher than in normal ones, and the expression went up over time (*P* < 0.01, Fig. 4b). Expression of HIF1A-AS2 was obviously up- or downregulated after transfection of pcDNA3.1-HIF1A-AS2 or sh-HIF1A-AS2 (*P* < 0.01, Fig. 4c); there was also an upward regulation of Runx2, Osterix, and Osteocalcin because of HIF1A-AS2 overexpression while HIF1A-AS2 silencing downregulated these markers (*P* < 0.05, *P* < 0.01, Fig. 4d, e). Alizarin red and ALP staining results indicated calcium nodule formation, and ALP activity was facilitated by HIF1A-AS2 overexpression and suppressed by HIF1A-AS2 silencing (*P* < 0.05, *P* < 0.01, Fig. 4f). These results showed that HIF1A-AS2 acted a positive part in ASC osteogenic differentiation.

RETRACTED

**Fig. 4:** Identification of ASCs and effect of HIF1A-AS2 on ASC osteogenic differentiation. **a** Flow cytometry for CD29/CD31/CD44/CD45 detection. **b** qRT-PCR: expression of HIF1A-AS2 in normal/induced ASCs over time. **c** qRT-PCR: expression of HIF1A-AS2 in induced ASCs after pcDNA3.1-HIF1A-AS2 or sh-HIF1A-AS2 transfection. **d** qRT-PCR: expression of Runx2, Osterix, and Osteocalcin after transfection. **e** Western blot analysis of Runx2, Osterix, and Osteocalcin after transfection. **f** Alizarin red staining (21 days) and ALP staining (14 days): changes of calcium nodule formation and ALP activity after transfection. ^*^P < 0.05, ^**^P < 0.01, compared with NC group; ^#^*P* < 0.05, ^##^*P* < 0.01, compared with sh-NC group

### HIF1A-AS2 regulated ASC osteogenic differentiation through miR-665

Expression of miR-665 was lower in induced ASCs and downregulated over time (*P* < 0.01, Fig. 5a). Dual-luciferase assay confirmed the predicted targeting relationship between miR-665 and HIF1A-AS2 (Fig. 5b) wherein co-transfection of wt HIF1A-AS2 3′UTR and agomiR-665 significantly reduced luciferase activity (*P* < 0.01, Fig. 5c). Transfection of agomiR-665 or antagomiR-665 notably facilitated or suppressed miR-665 expression, while the effects were neutralized by HIF1A-AS2 overexpression or silencing (*P* < 0.01, Fig. 5d). Expression of Runx2, Osterix, and Osteocalcin also reduced after transfection of agomiR-665 while antagomiR-665 brought an opposite effect (*P* < 0.05, *P* < 0.01, Fig. 5e, f). Alizarin red and ALP staining indicated that agomiR-665 suppressed calcium nodule formation and ALP activity, but antagomiR-665 or HIF1A-AS2 overexpression could reverse the process (*P* < 0.01, Fig. 5g).

RETRACTED

**Fig. 5:** Targeting relationship between HIF1A-AS2 and miR-665 and their effects on ASCs. **a** qRT-PCR: expression of miR-665 in normal/induced ASCs over time. **b** Predicted binding site between miR-556 and wt/mut HIF1A-AS2 3′UTR. **c** Dual-luciferase assay: luciferase activity in wt HIF1A-AS2 3′UTR + agomiR-665 group was significantly lower than that in wt HIF1A-AS2 3′UTR + agomiR-NC group. **d** qRT-PCR: expression of miR-665 in induced ASCs after agomiR-665, antagomiR-665, pcDNA3.1-HIF1A-AS2, or sh-HIF1A-AS2 transfection. **e** qRT-PCR: expression of Runx2, Osterix, and Osteocalcin after transfection. **f** Western blot analysis of Runx2, Osterix, and Osteocalcin after transfection. **g** Alizarin red staining (21 days) and ALP staining (14 days): changes of calcium nodule formation and ALP activity after transfection. ^*^P < 0.05, ^**^P < 0.01, compared with NC group; ^#^*P* < 0.05, ^##^*P* < 0.01, compared with sh-NC group

### MiR-665 regulated ASC osteogenic differentiation through IL6

Similar to HIF1A-AS2, IL6 was observed to be highly expressed in induced ASCs and upregulated over time (*P* < 0.01, Fig. 6a). Moreover, agomiR-665 could remarkably suppress IL6 expression, while antagomiR-665 had a reverse effect (*P* < 0.05, Fig. 6b). Dual-luciferase assay verified the target relationship between miR-665 and IL6 (Fig. 6c); co-transfection of agomiR-665 and wt IL6 3′UTR could prominently reduce luciferase activity (*P* < 0.01, Fig. 6d). The impact of agomiR-665 on Runx2, Osterix, and Osteocalcin expression can also be overturned by IL6 (*P* < 0.05, *P* < 0.01, Fig. 6e, f). Alizarin red and ALP staining displayed a similar result that IL6 could neutralize the impact of miR-665 on calcium nodule formation and ALP activity (*P* < 0.01, Fig. 6g).

**Fig. 6:** Targeting relationship between miR-665 and IL6 and their effects on ASCs. **a** qRT-PCR: expression of IL6 in normal/induced ASCs over time. **b** qRT-PCR: expression of IL6 in induced ASCs after agomiR-665, antagomiR-665, pcDNA3.1-IL6, or sh-IL6 transfection. **c** Predicted binding site between miR-556 and wt/mut IL6 3′UTR. **d** Dual-luciferase assay: luciferase activity in wt IL6 3′UTR + agomiR-665 group was significantly lower than that in wt IL6 3′UTR + agomiR-NC group. **e** qRT-PCR: expression of Runx2, Osterix, and Osteocalcin after transfection. **f** Western blot analysis of Runx2, Osterix, and Osteocalcin after transfection. **g** Alizarin red staining (21 days) and ALP staining (14 days): changes of calcium nodule formation and ALP activity after transfection. ^*^P < 0.05, ^**^P < 0.01, compared with NC group; ^#^*P* < 0.05, ^##^*P* < 0.01, compared with sh-NC group

RETRACTED

### HIF1A-AS2/miR-665/IL6 axis jointly regulated the PI3K/Akt signaling pathway

PI3K inhibitor LY294002 (10 μM) was applied to explore the impact of HIF1A-AS2/miR-665/IL6 on the PI3K/Akt signaling pathway. According to the result of western blot, overexpression of HIF1A-AS2/IL6 facilitates expression of protein IL6R which was the upstream protein of PI3K, Akt, and phosphorylated Akt (p-Akt), whereas agomiR-665 hinders their expression (*P* < 0.05, *P* < 0.01, Fig. 7a, b), indicating that HIF1A-AS2 might sponge miR-665, thus upregulating IL6, and high expression of IL6 leads to the PI3K/Akt signaling pathway activation. Enhancive calcium nodule formation and ALP activity was found when HIF1A-AS2/IL6 were overexpressed and agomiR-665/LY294002 groups had reverse results, which validates our conclusion on the cellular level (*P* < 0.05, *P* < 0.01, Fig. 7c).

**Fig. 7:** Effects of HIF1A-AS2/miR-665/IL6 axis on the PI3K/Akt signaling pathway. **a**, **b** Western blot: effects of pcDNA3.1-HIF1A-AS2/pcDNA-IL6/agomiR-665 and PI3K inhibitor LY294002 (10 μM) on expression of PI3K/Akt-related proteins IL6/IL6R/Akt/p-Akt, reflecting the activation of the PI3K/Akt signaling pathway. **c** Alizarin red staining (21 days) and ALP staining (14 days): changes of calcium nodule formation and ALP activity after pcDNA3.1-HIF1A-AS2/pcDNA3.1-IL6/agomiR-665 transfection or LY294002 treatment. ^*^P < 0.05, ^**^P < 0.01, compared with NC group; ^#^*P* < 0.05, ^##^*P* < 0.01, compared with sh-NC group

## Discussion

Statistical analysis and experiment results verified that lncRNA HIF1A-AS2 and mRNA IL6 were highly expressed in osteogenic induced ASCs, while knockdown of HIF1A-AS2/IL6 reduced osteoblast markers Runx2, Osterix, and Osteocalcin and impaired the osteogenic function. On the molecular level, HIF1A-AS2 sponged on miR-665, leading to IL6 increase and activation of the PI3K/Akt signaling pathway.

Recently, adipose-derived stem cells (ASCs) have gained extensive attention on their application in tissue engineering [33]. Scientists argued ASCs’ own multipotential in differentiation [3]; apart from adipose cells, they can also play a role in angiogenesis and soft tissue regeneration [34, 35], and as a prospective alternative autologous cell-based therapy to bone marrow stem cells [36], ASC transplant has been successfully applied in bone regeneration [37]. Evidence suggested that ASCs were analogous to BMSCs in many characteristics: morphology, transcriptome profiles, immunophenotype, and multilineage differentiation function [38–40]. By contrast, ASCs possess easier accessibility due to the abundance in the body, and less-invasive extraction procedures, lower incidence rate, and relatively low cost expand the advantage. In this study, we found a brand new chain which could accelerate the ASC osteogenic process.

RETRACTED

HIF1A-AS2 has already been found upregulated in some cancers; its influence on maintenance of mesenchymal glioblastoma stem-like cells is noteworthy [11]. Chen et al. revealed that HIF1A-AS1 and HIF1A-AS2 took part in periodontal ligament cell (PDLC) osteogenic differentiation which was regulated by hypoxia-inducible factor-1α (HIF-1α) [15]. It was primarily proved that HIF1A-AS1 played a role in PDLC osteogenic differentiation and it still needed further research in ASCs. In our research, HIF1A-AS2 and IL6 were found both upregulated in osteogenic cells through bioinformatics analysis. Besides, we found binding sites between HIF1A-AS2 and miR-665, and miR-665 could target IL6 by establishing sequence-specific interaction based on high-level consistency with 3′UTR, which indicated the upstream role of HIF1A-AS2 in the whole regulation process by sponging miR-665 to affect IL6 expression. It was reported HIF1A-AS2 could promote angiogenesis of the human umbilical vein endothelial cell by sponging to miRNA [14] and this regulation mode was consistent with the direction of our research. Heair et al. discovered that miR-665 functioned as a repressor of odontoblast maturation and mineralization by directly repressing the expression of the transcription factor Dlx3 and thus its downstream targets [24]. This was consistent with the inhibition of osteogenic differentiation by miR-665 in our experimental results.

Interleukin-6 (IL6) is a cytokine that stimulates the growth and differentiation of B lymphocytes and is also a growth factor for hybridomas and plasmacytomas. It is produced by many different cells including T lymphocytes, monocytes, and fibroblasts and concerns a variety of pathological and physiological processes [41]. Particularly, IL6 plays a crucial part in keeping the dynamic equilibrium between osteogenesis and bone resorption [42], and IL6 excreted by osteoblasts promotes osteoclast differential activities [43]. It is also reported that IL6 produced by adipose-derived stromal cells increases on account of the regulation of upstream factors and promotes the osteogenic differentiation of ASCs [44]. As an extensively researched signaling pathway, PI3K/Akt has been verified to be related to ossification [45, 46]. Our experiment results showed the level of IL6 increased in osteogenic-induced ASCs and activated the PI3K/Akt signaling pathway which contains an IL6 receptor, hence further promoting osteogenic differentiation. These results were in accord with previous reports.

RETRACTED

## Conclusions

In conclusion, the present work found out the regulatory mechanism of HIF1A-AS2/miR-665/IL6 axis via the PI3K/Akt signaling pathway in ASC osteogenic differentiation. HIF1A-AS2 was upregulated in induced ASCs, strengthening the miR-665 sponge, thereby promoting the expression of the target gene IL6 through activating the PI3K/Akt signaling pathway. This study provided a new idea for exploring new methods in stimulating ASC osteogenic induction and may be conducive for the development of tissue engineering and treatment for bone diseases and injuries.

## Additional file

Additional file 1: **Table S1.** KEGG pathway information of human. (DOCX 77 kb)

## Abbreviations

3′UTR: 3′-Untranslated regions
ALP: Alkaline phosphatase
ASCs: Adipose-derived stem cells
AVICs: Aortic valve interstitial cells
BMSCs: Bone marrow mesenchymal stem cells
BSA: Bovine serum albumin
ceRNA: Competing endogenous RNA
FBS: Fetal bovine serum
GEO: Gene Expression Omnibus
GSEA: Gene Set Enrichment Analysis
IL6: Interleukin-6
IL6R: IL6 receptor
KEGG: Kyoto Encyclopedia of Genes and Genomes
lncRNAs: Long noncoding RNAs
miRNAs: MicroRNAs
mRNA: Messenger RNA
MSC: Mesenchymal stem cell
PDLCs: Periodontal ligament cells
SD: Standard deviation
wt: Wild type
